# From Iron Metabolism to Ferroptosis: Pathologic Changes in Coronary Heart Disease

**DOI:** 10.1155/2022/6291889

**Published:** 2022-08-10

**Authors:** Xinbiao Fan, Aolin Li, Zhipeng Yan, Xiaofei Geng, Lu Lian, Hao Lv, Dongjie Gao, Junping Zhang

**Affiliations:** ^1^First Teaching Hospital of Tianjin University of Traditional Chinese Medicine, Tianjin 300183, China; ^2^National Clinical Research Center for Chinese Medicine Acupuncture and Moxibustion, Tianjin 300193, China

## Abstract

Coronary heart disease (CHD) is closely related to oxidative stress and inflammatory response and is the most common cardiovascular disease (CVD). Iron is an essential mineral that participates in many physiological and biochemical reactions in the human body. Meanwhile, on the negative side, iron has an active redox capacity, which leads to the accumulation of reactive oxygen species (ROS) and lipid peroxidation. There is growing evidence that disordered iron metabolism is involved in CHD's pathological progression. And the result of disordered iron metabolism is associated with iron overload-induced programmed cell death, often called ferroptosis. That features iron-dependent lipid peroxidation. Ferroptosis may play a crucial role in the development of CHD, and targeting ferroptosis may be a promising option for treating CHD. Here, we review the mechanisms of iron metabolism in cardiomyocytes (CMs) and explain the correlation between iron metabolism and ferroptosis. Meanwhile, we highlight the specific roles of iron metabolism and ferroptosis in the main pathological progression of CHD.

## 1. Introduction

Coronary atherosclerotic heart disease, also known as CHD, refers to localized myocardial ischemia, hypoxia, and even necrosis due to atherosclerosis (AS) [1]. As the population ages and people's lifestyles change, the morbidity and mortality of CHD are also increasing yearly. CHD is not only the most common CVD but also one of the leading causes of death worldwide [2]. And AS is the pathological basis of CHD, which involves inflammation, lipid deposition, plaque formation, and calcification. In addition, pathological changes such as vascular endothelial damage, arterial wall plaque stability damage, CM death, myocardial fibrosis (MF), and myocardial hypertrophy (MH) are also involved in the progress of CHD [3, 4].

Iron is an essential metal for the body and is the primary raw material for manufacturing hemoglobin and myoglobin. In addition, iron is critical for cellular viability and participates in a wide range of biochemical and physiological processes, including oxygen storage and transportation, mitochondrial respiration, DNA synthesis and repair, and enzymatic reactions in cells. However, excessive iron has toxic effects on the body. Iron has an active redox capacity, making it easy for free iron to receive and contribute electrons. The most important mechanism of iron biotoxicity is the involvement of excess intracellular ferrous iron (Fe^2+^) in the Fenton or Haber-Weiss reaction [5]. The interaction of Fe^2+^ with oxygen or hydrogen peroxide catalyzes the production of large amounts of ROS, leading to lipid peroxidation and further severe organ damage [6]. At the same time, Fe^2+^ is oxidized to ferric iron (Fe^3+^). Iron is also associated with the pathological mechanisms of various diseases such as hemochromatosis, cancer, and CVD [7, 8].

Recent studies have shown that dysregulation of iron metabolism is associated with CHD [9, 10]. Severe iron overload is involved in vascular injury and CM death, promoting the development of AS, myocardial infarction (MI), and heart failure (HF) [11]. And these results are related to iron overload-induced programmed cell death, or ferroptosis, a new form of programmed cell death discovered in recent years. Ferroptosis is featured by iron-dependent lipid peroxidation, unlike autophagy, apoptosis, and pyroptosis [12]. Some studies have directly or indirectly proved that ferroptosis exists in ischemic heart disease and plays an essential role in the process of CM death [13–15]. However, the effect of ferroptosis on CHD remains unclear. Here, we review the mechanisms of iron metabolism and regulation in CMs and explain the correlation between iron metabolism and ferroptosis. Moreover, we focus on the specific role of ferroptosis in the pathological progression of CHD.

## 2. Iron Homeostasis in CMs

Iron-mediated injury plays an essential role in many CVD, and studies on iron metabolism in the heart have attracted many scientists (Figure 1).

### 2.1. Iron Import in CMs

Systemic iron can form transferrin-bound iron (TBI) in the blood by binding to the transferrin (Tf), but binding sites in Tf have a limited high affinity for Fe^3+^. Studies have shown that the Tf saturation level is about 30% [16]. When high plasma iron concentration exceeds Tf iron binding capacity, iron mainly binds to serum albumin and citric acid to produce non-transferrin-bound iron (NTBI). TBI and NTBI both have access to CMs, but the pathways and regulatory mechanisms are different. CMs accumulate TBI through Tf receptors (TfRs), whereas accumulation of NTBI is via the divalent metal transporter 1 (DMT1), calcium channels, and zinc transporters.

#### 2.1.1. TBI-Dependent Pathways

Under physiological conditions, iron mainly combines with Tf and enters CMs through TfR1 on the cell membrane [17, 18]. Fe^3+^ is released in endosomes and then reduced to Fe^2+^ by the six-transmembrane epithelial antigen of prostate 3 (STEAP3). Subsequently, Fe^2+^ is transferred to the cytoplasm by DMT1. TfR1 gene has a conserved stem-loop structure in the 3′ untranslated region (UTR) called the iron response element (IRE). Iron regulatory protein (IRP) is the main protein that controls the balance of iron metabolism in CMs. IRP1 and IRP2, two forms of IRPs, have been found to act by binding to IRE [19]. The binding of IRP1 and IRP2 to IRE protected TfR1 mRNA from intranuclear degradation when CMs were iron deficient. That ensures the stability of TfR1 mRNA, increases its expression, and promotes iron absorption. Downregulation of TfR1 expression and a significant decrease in iron concentration occurred in mice with IRP gene knockout in CMs [20]. When iron overload occurs in CMs, IRP1 is converted to functional cytoplasmic aconitase via iron-sulfur clusters (Fe-S). At the same time, IRP1 loses its IRE-binding activity and the degradation of IRP2 increases. DMT mRNA with IRE in its 3′ UTRs has also been identified. IRE binding to IRP inhibits DMT mRNA degradation and facilitates iron uptake, which is consistent with the regulation of TfR1 [21].

#### 2.1.2. NTBI-Dependent Pathways

When iron overload occurs, plasma NTBI levels are elevated. There is a consensus that NTBI is potentially toxic and can cause tissue damage by increasing oxidative stress and inducing tissue iron overload. NTBI cannot enter cells through TfR1 but DMT1, L-type calcium channel (LTCC), T-type calcium channel (TTCC), zinc transporters, and other non-transferrin receptor-dependent pathways [22]. Studies have shown that LTCC and TTCC are the main pathways for NTBI to enter CMs. Efonidipine is a dual TTCC and LTCC blocker. In thalassemic mice, efonidipine reduced cardiac iron accumulation and improved cardiac function. However, it did not affect the expression of cardiac ferroportin (FPN) [23]. In addition, ZRT/IRT-like protein 14 (ZIP14) and DMT1 may be involved in the uptake of NTBI in CMs [20]. A vivo study found that ZIP14 is consistently expressed in iron overloaded hearts but is not upregulated in response to increased iron deposition. It is speculated that ZIP14 is involved in the uptake of NTBI by CMs, but there may be other pathways involved in the uptake of NTBI [24]. And the control of NTBI import by DMT1 is regulated by the IRP/IRE system. It should be noted that the entry of NTBI into CMs through calcium channels and zinc transporters is not affected by IRP/IRE, but the specific regulatory mechanism remains unclear.

### 2.2. Iron Export from CMs

Once iron enters CMs, it becomes part of the labile iron pool (LIP). Iron enters the mitochondria as a feedstock for heme and Fe-S. In addition, ferritin (FT) stores some of the iron, and FPN exports the excess iron. Iron can enter CMs through multiple pathways, but only FPN is the export pathway, suggesting that CMs are particularly sensitive to iron overload. One study specifically knocked out FPN in the hearts of mice and found that their cardiac function was severely impaired, which was associated with cardiac iron overload [9]. However, there was no significant change in systemic iron status, suggesting that CMs have their unique regulation mechanism of iron metabolism. Notably, IREs are also present in the 5′ UTR of FPN mRNA and FT mRNA. The combination of IRE and IRP inhibits the translation of FPN and FT and prevents intracellular iron export and storage. Another more critical mechanism of iron export regulation is the role of the hepcidin (HEP)-FPN axis in the heart. The HEP-FPN axis in the heart is not affected by systemic HEP. Myocardial iron deficiency or hypoxia promotes local HEP expression and limits iron export by degrading FPN [10, 25]. A study prepared mouse models of HEP-resistant FPN knockout and cardiomyocyte-specific deletion of HEP. Both models showed severe cardiac dysfunction and iron deficiency in CMs rather than systemic iron deficiency [26]. A recent study found that knock-in HEP-resistant FPN in mouse pulmonary arterial smooth muscle cells (SMCs) leads to pulmonary hypertension and HF, suggesting that the HEP-FPN axis also plays a crucial role in regulating vascular homeostasis [26].

## 3. Effect of Iron Accumulation on Cardiac Ischemic and Hypoxic Injuries

During the development of CHD, we can observe abnormalities in multiple cell death signaling cascades. These include apoptosis, autophagy, pyroptosis, and ferroptosis (Table 1). Disordered iron metabolism runs through the whole pathological progression of CHD, and iron overload is considered an essential pathological factor of cardiovascular injury [9]. The data suggested that nearly 1/3 of the iron in CMs is distributed in mitochondria, catalyzing electron transport through the reversible oxidation state of iron and providing the energy required for normal cardiac function. Mitochondrial function is associated with disordered iron metabolism in the development of CVD [27]. When myocardial ischemia and hypoxia occur, LIP is imbalanced. Iron overload leads to the peroxidation of oxygen radicals in the cytoplasm and mitochondria. And it then will damage DNA, proteins, and lipids, resulting in cardiotoxicity [27]. In addition, AS was shown to be exacerbated significantly in FPN knockout mice, suggesting that iron overload has a promotive effect on AS. This effect is associated with iron overload-induced pathological changes, including dyslipidemia, altered vascular permeability, sustained endothelial activation, and elevated proinflammatory mediators. However, iron clearance mediated by transferrin or iron chelators and a low-iron diet may rescue NTBI-mediated toxicity [28].

Iron metabolism and oxidative stress in CMs are closely related to autophagy. Autophagy is a process of cellular self-feeding that relies primarily on lysosomes for intracellular degradation and recycling, promoting cellular repair or accelerating cell death. Thus, autophagy plays a dual role in maintaining cellular homeostasis and promoting cell renewal and metabolism [29]. Autophagy is activated by various environmental stressors, such as energy depletion, nutrient deficiency, and endoplasmic reticulum stress [30]. Appropriate autophagy can protect CMs by reducing oxidative stress and weakening myocardial inflammation, but excessive autophagy can lead to CM death and thus aggravate cardiac functional impairment. In the early stage of myocardial ischemia and hypoxia, appropriate autophagy facilitates the removal of mitochondria from damaged tissues, reduces the production of ROS, and maintains CM homeostasis to protect the heart from ischemic injury. However, in the late phase of myocardial ischemia and hypoxia, disordered iron metabolism induces CM autophagy to release iron stored in FT [31]. In addition, ferritinophagy is mediated by NCOA4 and exacerbates myocardial injury by increasing cellular unstable iron levels through degradation of cellular FT and induction of TfR1 expression, which subsequently sensitizes cells to ferroptosis [32]. Erastin is a classical ferroptosis inducer that acts on multiple molecular structures to induce ferroptosis. According to published reports, NCOA4 can prevent erastin-induced ferroptosis [33]. Therefore, timely regulation of autophagic by maintaining iron homeostasis during myocardial ischemia and hypoxia can reduce autophagy-induced myocardial injury.

## 4. Effect of Iron and ROS on Ferroptosis in the Heart

Ferroptosis is a newly discovered form of regulated cell death driven by iron-dependent lipid peroxidation. A growing number of studies have demonstrated that lipid peroxidation is a key trigger and landmark event in ferroptosis [39]. And high levels of intracellular NTBI are a prerequisite for triggering ferroptosis [40]. Extensive ROS generated by intracellular iron via the Fenton reaction and the Haber-Weiss reaction can directly produce a chain reaction with polyunsaturated fatty acids (PUFAs) in membrane phospholipids [38]. Further analysis has shown that AA and AdA are essential phospholipids to facilitate the peroxidation reaction [41]. PUFAs are highly sensitive to lipid peroxidation due to their unstable double bonds. With the help of ACSL4 and LPCAT3, PUFAs in cell membranes undergo synthesis, activation, and incorporation into phospholipids to produce PUFA-phosphatidyl ethanolamine (PUFA-PE) [42]. That makes the cell membrane easier to be attacked by ROS and produces more lipid peroxides. Also closely associated with ferroptosis is lipoxygenase (LOX). It can catalyze the peroxidation reaction of PUFA-PE [42]. Harmful lipid peroxides are scavenged by the intracellular antioxidant system when they accumulate. However, when the antioxidant system is weakened, lipid peroxides will not be scavenged in time, leading to an attack on the cytoplasmic membrane and morphological changes associated with ferroptosis [43]. Notably, ferroptosis inhibitors has been proven to inhibit the occurrence of ferroptosis [15, 44]. Research has shown that MI can lead to high levels of ROS production in the myocardium and that ferrostatin-1 (Fer-1) can significantly reduce the area of MI [45].

## 5. Regulatory Pathways of Ferroptosis

Under physiological conditions, the antioxidant response in the body is in a relative balance. When this balance is disrupted, it causes the accumulation of free radicals and triggers ferroptosis [46]. The System Xc- glutathione (GSH)-glutathione peroxidase 4 (GPX4) axis is the central redox mechanism inhibiting ferroptosis [47]. GSH is an essential antioxidant in the oxidative stress response, and cystine is one of the basic raw materials for GSH synthesis. GPX4 is an antioxidant enzyme that scavenges lipid peroxides and prevents the conversion of iron-dependent conversion of lipid peroxides to more reactive lipid radicals [48]. The reduction of toxic lipid peroxides to nontoxic lipid alcohols by GPX4 depends on the electrons provided by GSH [43]. System Xc- is a cystine/glutamate antiporter composed of SLC7A11 and SLC3A2, which mediates the exchange of extracellular cystine with intracellular glutamate and is responsible for the transport of cystine into the cell [49]. When selectively inhibiting System Xc-, cystine uptake will be reduced, and GSH synthesis in the organism will also be reduced [50]. Notably, erastin causes GSH depletion and GPX4 inactivation by inhibiting System Xc-, inducing ferroptosis [51]. The expression of SLC7A11 and GPX4 was significantly decreased in H/R-induced H9C2 cells. In addition, the naringin ameliorated cardiomyocyte ferroptosis via the System Xc-/GPX4 axis. However, the protective effect could be counteracted by erastin [52]. The data confirmed that the System Xc-GSH-GPX4 axis plays an essential role in the process of myocardial injury.

In addition to the System Xc-GSH-GPX4 axis, several pathways of ferroptosis regulation have been identified (Figure 2). Among them, the GCH1-BH4 pathway and the FSP1-CoQ-NADPH pathway are the other two independent mechanisms unaffected by GPX4 [47]. BH4 is a potent antioxidant. The expression of GCH1 triggers the production of BH4, thus exerting an antioxidant effect to inhibit ferroptosis [53, 54]. CoQ10 is another strong oxidant, and its fully reduced state, CoQH2, can trap lipid peroxide radicals and prevent peroxidative damage to the plasma membrane. FSP1 is a novel oxygen reductase that inhibits ferroptosis. It can catalyze CoQ10 regeneration dependent on NADPH and inhibit GPX4 deficiency-induced ferroptosis [55, 56].

## 6. Ferroptosis Involvement in the Pathological Progression of CHD

The primary pathological mechanism of CHD lies in the formation, growth, and even rupture of atherosclerotic plaques, resulting in luminal narrowing or blockage. Reduced myocardial perfusion induces MI and eventually leads to the progression of HF [3]. Several studies have shown that iron metabolism and ferroptosis are involved throughout the development of CHD and influence the key pathological changes of CHD. These include vascular endothelial damage, arterial wall plaque stability damage, CM death, MF, and MH [11, 37] (Table 2).

### 6.1. Vascular Endothelial Damage

Vascular endothelial cells (VECs) are border cells between blood and the vascular wall. They have highly selective permeability and are biological barriers to the interchange of material and protection of the inner surface of blood vessels [74]. Normal VECs have the effects of regulating vascular tone, procoagulation, antithrombosis, and anti-inflammatory, which are critical for maintaining vascular homeostasis [75]. VEC dysfunction and morphological damage are the beginning of AS and participate in the occurrence and development of CHD. In the early stages of AS, risk factors lead to increased adhesion molecule expression and dysregulation of antioxidant effects [76, 77]. All these alterations lead to the adhesion of leukocytes (especially monocytes) to VECs. Monocytes adhering to the vascular intima gradually migrate to the intima and differentiate into macrophages in response to inflammatory factors and the expression of receptors that facilitate lipid uptake [78]. As a result, lipid components of the blood, especially low-density lipoprotein (LDL), are absorbed and gradually deposited in the intima. LDL is oxidatively modified to oxidize LDL (ox-LDL) in the subintima. The oxidative process and toxic effects of ox-LDL can lead to or aggravate vascular endothelial damage and dysfunction, thereby significantly promoting lipid deposition [79]. Subsequently, scavenger receptors on the surface of macrophages can rapidly recognize ox-LDL and phagocytose it to form foam cells. Foam cells and lipids accumulate massively under the intima, producing an early lesion of AS known as fatty streaks [80, 81].

Although the pathological mechanism of AS is complex, current studies emphasize that oxidative stress is a key factor in the occurrence and development of AS. ROS generated during oxidative stress can oxidize lipids and proteins, induce inflammatory responses, and directly damage vascular cells, leading to endothelial dysfunction [82, 83]. Iron is considered potentially toxic because of its intense oxidative activity. When iron is overloaded, the body can produce large amounts of oxygen free radicals that injure VECs and other target cells [6, 84]. FPN is the only pathway of iron export in cells. If FPN is lost, intracellular and systemic iron overload will occur [9]. In one study, deletion of apoE and FPN genes in mice led to increased NTBI and induced chronic iron overload, subsequently increasing vascular oxidative stress levels and promoting AS [28]. These results may result from iron overload-induced endothelial activation and dysfunction. In contrast, restricting dietary iron intake or treating with iron chelators inhibited the progression of AS in mice [28].

The imbalance of redox reactions and iron overload as the main characteristics of ferroptosis provide indirect evidence to explore the role of ferroptosis in vascular endothelial damage in AS [85]. Direct evidence suggested that VEC ferroptosis was observed in diabetic AS mouse models [57]. The mice showed iron overload, downregulation of GPX4, and lipid peroxidation following upregulation of HMOX1. In addition, the study also found that Fer-1 alleviated the increase in ROS and endothelial dysfunction induced by a high-fat-high-sugar diet [57]. Ox-LDL is commonly used to prepare animal models of AS, and multiple studies have found that AS induced by ox-LDL is associated with ferroptosis [60, 63]. The prenyldiphosphate synthase subunit 2 (PDSS2) is a primary regulator of AS [86]. In ox-LDL-induced human coronary AS models, PDSS2 inhibited VEC ferroptosis and AS progression by promoting Nrf2 activation, thereby inducing the proliferation of human coronary endothelial cells [58]. Research has shown that miR-17-92 protected VECs from erastin-induced ferroptosis by targeting the A20-ACSL4 axis [59]. As a classical lipid-lowering drug, fluvastatin reversed the reduction of GPX4 and xCT levels induced by ox-LDL, thus achieving inhibition of VEC ferroptosis and vascular protection [60]. The discovery provides scientific evidence for the new role of statins in the prevention and treatment of AS. In terms of environment and health, studies have shown that PM2.5 accelerates the progression of CVD in numerous ways [87]. A recent study showed that PM2.5-induced vascular endothelial damage is also associated with ferroptosis [40]. The data showed that PM2.5 increases ROS production and iron content in VECs. In addition, the study provided the primary evidence for ferroptosis induced by iron uptake and storage dysfunction (disordered iron metabolism) by monitoring transferrin receptor, ferritin light chain (FTL), and ferritin heavy chain (FTH1) expression. This study further found that PM2.5 decreased the levels of GSH, glutathione peroxidase (GSH-Px), and NADPH. It was concluded here that PM2.5 induces VEC ferroptosis [40]. Although the mechanism of vascular endothelial damage is still unclear, the role of ferroptosis in triggering endothelial dysfunction has been widely proved. And Fer-1 and iron chelators can reverse the toxicity to a certain extent. Therefore, exploring the relationship between ferroptosis and endothelial damage is relevant to the mechanism research and prevention of CHD.

### 6.2. Arterial Wall Plaque Stability Damage

With the development of coronary AS, macrophages constantly phagocytize lipids and transform them into foam cells. At the same time, macrophages secrete inflammatory cytokines, which aggravate the local inflammatory response and further promote macrophage death [88]. That will further accelerate the formation of plaques and destabilize them. Under the stimulation of inflammation, SMCs in the middle membrane of the coronary artery migrate to the intima. Subsequently, they fuse with SMCs in the intima, proliferate, and secrete extracellular matrices (ECMs), such as elastin and interstitial collagen. SMCs and ECMs are the main components of the fibrous cap. They cover the foam cells and lipids accumulated under the intima. Then, the lipid core of the plaque gradually forms [89]. Under the stimulation of long-term hypoxia and inflammation, foam cells in the lipid core die in various ways and release lipids and cell debris. Significant amounts of cell components accumulate in the central area of plaques, forming a lipid-rich pool called the necrotic core [90]. As the pathological basis of coronary atherosclerotic plaque formation, necrotic core and fibrous cap are closely related to the unstable progress of the plaque. Angina pectoris occurs when the coronary arteries gradually narrow with plaque growth and block the blood supply to the heart muscle. When acute thrombosis obstructs large coronary vessels, blood flow is rapidly interrupted, leading to MI and unstable angina [91]. The foremost common cause of thrombosis is the rupture of vulnerable plaques. It has been established that the characteristics of vulnerable plaques include massive monocyte/macrophage infiltration, bulky lipid-rich necrotic cores, thin fibrous caps, and fewer SMCs [92]. Macrophages under the fibrous cap can reduce ECMs by their phagocytic function. The macrophages also can secrete plenty of matrix metalloproteinases to hydrolyze ECMs within the fibrous cap. As a result, the fibrous cap becomes thin and brittle, causing the plaque to become unstable and rupture to form a thrombus [80, 93]. In contrast, SMCs can secrete ECMs, which are the main ingredient of the fibrous cap, thus improving plaque stability [89]. Therefore, understanding further the role of macrophages and SMCs in plaque stability may provide new ideas for treating CHD.

Recent studies have shown that increased free iron can promote pathological processes such as oxidative stress and lipid peroxidation, accelerating inflammation and the formation of macrophage-derived foam cells, thus affecting plaque stability [61]. There are two primary sources of reactive iron in atherosclerotic plaques. One is plaque rupture and bleeding, and the other is the phagocytosis and rapid lysis of red blood cells by macrophages [94]. Considering the significant role of macrophages in systemic iron metabolism and the formation and progression of atherosclerotic plaques, Apoe^−/−^ mouse models of macrophage-specific FPN1 deficiency were prepared in a study to investigate the effects and mechanisms of iron overload in macrophages on the progression of CHD [62]. The results indicated that iron overload in macrophages inhibited ATP-binding cassette (ABC) transporter protein expression by downregulating the liver X receptor *α* (LXR*α*) expression. This progression increased oxidative stress and systemic inflammation levels, promoted foam cell formation, and restricted lipid efflux, ultimately contributing to AS progression. In addition, iron overload also causes several changes in the composition of atherosclerotic plaques, with an increase in the number of macrophages and a decrease in collagen within the plaques, which make the plaques more prone to rupture [62]. However, iron chelation therapy increased ABC transporter protein expression, reversed lipid deposition, and reduced the surface volume of atherosclerotic plaques, ultimately slowing the progression of AS [62]. In another study, high levels of uric acid inhibited the Nrf2/PTGS2/GPX4 signaling pathway, induced the formation of macrophage-derived foam cells, and lipid peroxidation, thereby promoting the progression of AS. However, all these changes were reversed by Fer-1 [63]. There are no systematic studies to explore the mechanism between macrophage ferroptosis and CHD. Even so, several studies have shown that ROS accumulation, lipid oxidation, and iron deposition in macrophages are critical features of advanced atherosclerotic plaques [95]. Thus, macrophage ferroptosis may play an essential role in coronary AS and vulnerable plaque formation. And regulation of macrophage ferroptosis may be a promising approach to enhance plaque stability and delay the progression of CHD.

Unlike macrophages, SMCs impair the stability of atherosclerotic plaques mainly by affecting fibrous cap components [89]. A study found that iron overload stimulated SMCs to migrate, proliferate abnormally, and calcify, causing them to acquire a macrophage-like phenotype. In addition, iron overload increased ROS production to create a prooxidant microenvironment, which promoted foam cell formation and plaque instability progression. Moreover, researches demonstrated that removing excess iron and reducing the production of ROS can reverse these results mentioned above [96–98]. Notably, cigarettes are a major risk factor for AS. A study found that cigarette smoke extract (CSE) induced ferroptosis in vascular SMCs but not VECs [64]. The data showed increased PTGS2 expression, GSH depletion, and lipid peroxidation in vascular SMCs. However, GPX4 overexpression had no significant effect on CSE-induced ferroptosis [64]. The triggering mechanisms of ferroptosis in SMCs and VECs may be different. Therefore, inhibiting ferroptosis in SMCs may also be a new research direction for plaque stabilization.

### 6.3. Cardiomyocyte Death

The main pathological change of CHD is the formation and development of atherosclerotic plaques. The plaques gradually increase in size or even fall off, narrowing or blocking the lumen of the arterial blood vessels, resulting in insufficient blood supply to the coronary arteries. And the lack of perfusion causes local damage and mass death of CMs [99]. CMs are terminally differentiated cells with extremely limited regenerative capacity [100]. The mass death of CMs will result in structural and functional defects in the heart and cause HF [101]. The best way to prevent ischemic damage to the heart is to restore blood flow to the myocardial tissue, also known as reperfusion. However, reperfusion itself can also cause damage to the myocardium, called myocardial ischemia/reperfusion (I/R) injury. The mechanisms involved are oxidative stress, calcium overload, and mitochondrial damage, all of which can cause CM death [102]. Therefore, how to prevent CM death is key to improving and restoring cardiac function after MI and myocardial I/R injury. New insights into how cells are programmed to die have provided new ideas for salvaging myocardial injury in recent years. A study showed increased iron deposition and ROS in CMs around the MI region during ischemia and early reperfusion, suggesting that ferroptosis is a prominent form of CM death [103].

In HF mouse and rat models after MI, FTH levels were significantly downregulated, and oxidative stress and free iron levels were significantly increased. And then, desferrioxamine, an iron chelator, reversed these results and improved the viability of CMs [14]. Iron overload as a crucial mechanism for ferroptosis occurrence has attracted scientists to explore the underlying mechanisms of ferroptosis involvement in CM death. Either erastin or isoproterenol-treated H9C2 cells significantly increased free iron levels and promoted lipid peroxidation, thereby decreasing the viability of CMs. This result suggested that ferroptosis is associated with CM death. Both Fer-1 and puerarin upregulated the expression of GPX4 and FTH1 and inhibited ferroptosis [65]. In another study, the levels of GPX4 protein and GPX4 mRNA expression were downregulated in mice during early and midstage MI. To further determine the role of GPX4 in CM ferroptosis, a study transfected H9C2 cells with GPX4 siRNA. The results showed a significant increase in malondialdehyde (MDA) and superoxide dismutase (SOD) levels. And Fer-1 reduced CM death induced by GPX4 downregulation and inhibited lipid peroxide production, which suggested that ferroptosis is involved in CM death and myocardial injury after MI and is partially associated with reduced GPX4 levels [66]. In addition, studies have demonstrated that NADPH oxidase (NOX), a key enzyme for ROS production, is highly expressed in CMs [104]. In the descending aortic banding procedure-induced HF models, ferroptosis and autophagy were associated with massive CM death, and they were regulated by the TLR4-NOX4 pathway. It mainly showed downregulation of TLR4 and NOX4 expression, decreased LC3B-II and Belcin1, and upregulation of p62, GPX4, and FTH1 protein expression. It also significantly reduced CM death and improved cardiac function [69]. Drugs targeting the associated pathways of autophagy and ferroptosis in CMs may also be new therapeutic strategies for CHD, but others in both need to be studied in depth. Currently, CM ferroptosis during MI and HF has not been well studied. Are these mechanisms still applicable to clinical practice? Is blocking the process of ferroptosis in CMs effective? Addressing these questions may lead to new treatments to protect CMs from ferroptosis and delay the progression of MI to HF.

The exosome of MSCs derived from HUCB-MSC is known to alleviate myocardial injury caused by MI in mice. In the CM H/R models, investigators found that overexpression of DMT1 promoted CM ferroptosis. However, HUCB-MSC exosomes could inhibit H/R-induced CM ferroptosis through the miR-23a-3p/DMT1 axis and attenuate myocardial injury [13]. In addition, dexmedetomidine was demonstrated to inhibit myocardial I/R-induced ferroptosis via the SLC7A11/GPX4 axis [67]. Iron overload and ferroptosis have also been found in myocardial I/R. In one study, propofol inhibited ferroptosis via the AKT/P53 signaling pathway, thereby protecting CM from I/R injury. Specifically, it reduced SOD and iron accumulation, decreased lipid peroxidation levels, thereby increasing the expression of antioxidant enzymes [68]. Ferroptosis as one of the mechanisms of CM death after myocardial I/R has been widely demonstrated, and inhibiting ferroptosis may be an effective way to attenuate myocardial I/R injury.

### 6.4. Myocardial Fibrosis

MF after MI is a process of self-repair and inflammatory response of the myocardium [105]. The pathology is characterized by the proliferation of myofibroblasts in the myocardial tissue, secretion and excessive deposition of ECMs, and disorders in the ratio and arrangement of various types of collagen [106, 107]. After MI, local ischemia and hypoxia lead to the mass death of CMs. The body then produces a repair response that includes cardiac fibroblast activation, proliferation, and phenotypic transformation to form myofibroblasts. The above pathological changes lead to a replacement fibrotic process, in which fibroblasts and myofibroblasts produce fibrous scars to replace the damaged tissue [108]. Furthermore, the process of replacement fibrosis will reduce further dilatation of the infarcted area and maintain the structural integrity of the ventricles, thus preventing cardiac rupture. In addition, increased intraventricular mechanical pressure and inflammatory response after MI can induce expansion of connective tissue in the noninfarcted region and cause reactive fibrosis in the noninfarcted area. Reactive fibrosis can alter ventricular compliance and increase ventricular wall stiffness, thus affecting cardiac systolic and diastolic function and synchronicity, eventually leading to HF, worsening arrhythmias, and even sudden death [106, 109]. MF is a significant manifestation of cardiac remodeling and an essential factor influencing the prognosis of MI. Therefore, inhibition of the progression of reactive fibrosis in the peripheral myocardium of the infarct area would be an ideal treatment after MI.

In one study, iron overload increased oxidative stress levels and led to MF in gerbil hearts, as evidenced by increased MDA levels and decreased GPX4 levels [70]. It is suggested that iron overload may foster MF development by inducing lipid peroxidation damage. In addition, GPX4 participates in various pathological processes such as inflammation, cellular repair, oxidative stress, and ferroptosis. And GPX4 is closely associated with the development of fibrotic diseases [48]. Recent studies on ferroptosis intervention in MF have focused on GPX4. In myocardial I/R injury mouse models, miR-375-3p was found to promote MF development by downregulating GPX4 expression. However, both miR-375-3p inhibitors and Fer-1 significantly attenuated MF in these mice and enhanced the antioxidant capacity of cardiac fibroblasts in vitro [71]. In another study, dexmedetomidine activated the SLC7A11/GPX4 signaling pathway, inhibited CM ferroptosis after myocardial I/R in mice, and significantly reduced the area of MF. Predictably, the extent of myocardial injury and fibrosis area markedly increased following erastin treatment [67]. All these studies have confirmed the role of ferroptosis in MF. However, the current studies on its pathogenesis are relatively homogeneous, without distinguishing the location and type of MF occurrence. Future studies should delve into the effects of ferroptosis on reactive fibrosis and its mechanisms.

### 6.5. Myocardial Hypertrophy

CHD, especially MI, leads to CM damage or death due to ischemia and hypoxia, resulting in a localized cardiac function deficit. Under prolonged stimulation, peripheral CMs gradually hypertrophy to compensate for partial cardiac function [110, 111]. The early stage of MH is a beneficial compensatory response for the organism, but its compensatory capacity is limited. The late-stage shows increased myocardial oxygen consumption and reduced cardiac compliance and contractility, leading to loss of compensatory effect of pathological MH, further increasing the risk of HF and malignant arrhythmias [112, 113]. Studies have shown that MH is an independent risk factor for increased morbidity and mortality from various CVD during clinical practice [114, 115].

Apelin-13 can accelerate the progression of MH. In a study, apelin-13 induced hypertrophy and elevated free iron levels in H9C2 cells. It was further observed that apelin-13 increased iron and ROS levels in mitochondria of CM and triggered mitochondrial damage. This experiment showed that apelin-13-stimulated MH was closely related to NCOA4-mediated ferritinophagy and sideroflexin 1 (a mitochondria iron transporting protein) mediated mitochondrial iron overload [72, 116]. The initial relationship between ferroptosis and MH has also been established. In addition, one study used angiotensin II to induce MH in mice and found that oxidative stress and ferroptosis occurred [50]. Knockdown of xCT increased PTGS2, MDA, and ROS levels and exacerbated Ang II-induced MH in mice [50]. In addition, Beclin 1 is a homolog of the yeast autophagy gene Atg6/Vps30, an essential molecule in the autophagic process. A study found elevated levels of SLC7A11, GPX4, and NCOA4 in Beclin 1 haploinsufficient mice. They promoted autophagy and ferroptosis and exacerbated low-temperature-induced MH [73]. Currently, there is no direct evidence that post-MI ferroptosis is associated with MH. However, MH induced by other methods is strongly associated with iron overload and ferroptosis. These studies further imply the potential of ferroptosis as a therapeutic target for MH after MI.

## 7. Ferroptosis as a Novel Therapeutic Target for CHD

As discussed above, ferroptosis has been found to play a significant role in the pathological progression of CHD [11, 37]. Accordingly, targeting ferroptosis will become a new therapeutic strategy for treating CHD. With intensive studies on the mechanisms and regulatory pathways of ferroptosis, three main methods of ferroptosis inhibition have been identified.

First, iron chelators can bind to iron in the body to effectively increase iron excretion, thus blocking the redox reaction caused by iron overload. Currently, the main iron chelators used in clinical practice are deferoxamine, deferiprone, and deferasirox [117]. Several studies have shown that iron chelators have cardiovascular protective effects, such as improving vascular endothelial function, inhibiting SMC proliferation, and protecting CMs [64, 118]. Second, genetic manipulation of ferroptosis has been shown to inhibit ferroptosis and reduce myocardial injury [119]. These include upregulation of GPX4 and overexpression of SLC7A11 [66, 120]. However, this approach is currently not clinically applicable. Last, the cardioprotective effects of antioxidants have also been widely demonstrated [121]. Fer-1 is one of the most common antioxidants. It can upregulate the expression of GPX4 and FTH1, thus inhibiting lipid peroxidation [65]. And Fer-1 can slow down the progression of AS and reduce the area of MI [45, 57, 63]. Vitamin E is a common clinical antioxidant that can inhibit ferroptosis by inhibiting LOX [41]. Therefore, antioxidants may be the most promising ferroptosis inhibitors for widespread use. Excavating drugs with inhibiting ferroptosis from clinically available drugs may provide new options for treating CHD more quickly, such as vitamin E, fluvastatin, puerarin, dexmedetomidine, and propofol [41, 60, 65, 67, 68].

## 8. Conclusions

This article reviews the mechanisms of iron metabolism in CMs. It also focuses on the role of iron metabolism and ferroptosis in the crucial pathological changes of CHD. In contrast, the current research on the mechanisms of ferroptosis is still at an early stage, and most findings are obtained from animal and cellular experiments. We cannot conclude whether inhibition of ferroptosis is totally beneficial at different stages of human CHD. Inhibition of vascular and cardiac ferroptosis may bring new benefits to patients with CHD. Therefore, exploring the mechanisms and clinical feasibility is necessary for future studies. At this point, we have some unanswered questions that need to be concerned. (1) What are the roles and mechanisms of iron overload and ferroptosis in intraplaque angiogenesis? (2) Is ferroptosis involved in cardiomyocyte proliferation a target for cardiac regeneration? (3) How do we select methods to regulate ferroptosis in the pathological progression of CHD? With ongoing research, the mystery of ferroptosis will be further uncovered. Maintaining iron homeostasis and targeting ferroptosis will be promising strategies for the staged treatment of CHD.

## Figures and Tables

**Figure 1:** Iron homeostasis in cardiomyocytes. TBI enters cardiomyocytes via TfR1. TBI is reduced to Fe^2+^ by STEAP3 after release in the endosome, and Fe^2+^ is transferred to the cytoplasm by DMT1. NTBI enters via DMT1, LTCC, TTCC, and ZT. After entering the CMs, iron becomes part of the LIP and works through different pathways. A portion of iron is used by mitochondria to produce heme and Fe-S, and a portion is stored in FT. Furthermore, another part of iron is exported through the FPN and regulated by HEP. And cardiac iron homeostasis is regulated by IRP-IRE. TBI: Tf-bound iron; NTBI: non-Tf-bound iron; TfR1: transferrin receptor 1; STEAP3: six-transmembrane epithelial antigen of prostate 3; DMT1: divalent metal transporter 1; LTCC: L-type calcium channel; TTCC: T-type calcium channel; ZT: zinc transporters; LIP: labile iron pool; FT: ferritin; FPN: ferroportin; Fe-S: iron–sulfur cluster; mtFT: mitochondrial ferritin; HEP: hepcidin; IRE: iron-responsive elements; IRP: iron regulatory protein.

**Figure 2:** The regulatory mechanisms of ferroptosis in the pathological progression of CHD. There are three major independent regulatory pathways of ferroptosis: the System Xc-GSH-GPX4 axis, the GCH1-BH4 pathway, and the FSP1-CoQ-NADPH pathway. In addition, iron metabolism and lipid peroxidation are the main mechanisms. Abbreviations: PUFAs: polyunsaturated fatty acids; PUFA-PE: polyunsaturated fatty acid-phosphatidyl ethanolamine; ACSL4: acyl-CoA synthetase long-chain family member 4; LPCAT3: lysophosphatidylcholine acyltransferase 3; LOX: lipoxygenase; SLC7A11: subunit solute carrier family 7 member 11; SLC3A2: solute carrier family 3 member 2; Glu: glutamate; GSH: glutathione; GPX4: glutathione peroxidase 4; GTP: guanosine triphosphate; BH4: tetrahydrobiopterin; GCH1: guanosine triphosphate cyclohydrolase 1; FSP1: ferroptosis suppressor protein 1; NCOA4: nuclear receptor coactivator 4; NADPH: nicotinamide adenine dinucleotide phosphate; ROS: reactive oxygen species; FT: ferritin; LIP: labile iron pool; CoQ10: coenzyme Q10.

**Table 1:** Comparison of different forms of programmed cell death.

Cell death mode	Morphological characteristics	Biochemical features	Characteristic molecules	References
Apoptosis	Chromatin condensation, nuclear fixation, cell shrinkage, membrane blistering, and formation of apoptotic bodies	DNA fragmentation, no leakage of cell contents, no inflammatory reaction	Caspase 3, caspase 7, caspase 8, BCL-2, Bax, P53, Fas	[34, 35]

Autophagy	Accumulation of double-membraned autophagic vesicles	Increased lysosomal activity	Beclin 1, mTOR, ATG5, ATG7, LC3, TFEB, DRAM-3	[35]

Pyroptosis	Nuclear consolidation, plasma membrane pore formation, cell swelling and rupture	DNA fragmentation and inflammatory cascade response	NLRP3, ASC, pro-caspase 1, IL-1*β*, IL-18	[4, 36]

Ferroptosis	Mitochondrial shrinkage, increased membrane density, decreased mitochondrial cristae, and outer membrane rupture	Iron overload, lipid peroxidation, mitochondrial membrane potential changes	ACSL4, LPCAT3, xCT, GPX4, Fer-1, OxPLs, TfR1, SLC7A11, Nrf2, NCOA4	[37, 38]

**Table 2:** Ferroptosis involvement in the pathological progression of CHD.

Histological type	Interventions	Features or changes	Pathways or signals	References
Vascular endothelial damage	Knock out FPN genes	Increase NTBI, induce chronic iron overload, increase vascular oxidative stress levels, promote AS		[28]
	High sugar and high lipid diet	Iron overload, elevated ROS level, downregulation of GPX4 and lipid peroxidation	HMOX1 increase	[57]
	PDSS2	Inhibit VEC ferroptosis and AS progression	Nrf2 activation	[58]
	miR-17-92 overexpression	Reduce erastin-induced growth inhibition and ROS generation of HUVEC	A20-ACSL4 axis	[59]
	Fluvastatin	Reverse ox-LDL-induced decreases in GPX4 and xCT levels	Regulate GPX4 and xCT	[60]
	PM2.5	Increase ROS production and iron content, decrease GSH, GSH-Px, and NADPH levels, promote lipid peroxidation		[40]

Arterial wall plaque stability damage	High-iron diet	Iron overload, accelerate inflammation and the formation of macrophage-derived foam cells		[61]
	Macrophage-specific FPN1 deficiency	Iron overload, increase oxidative stress and systemic inflammation levels, inhibit ABC transporter protein expression, increase numbers of macrophages, decrease collagen	Downregulate LXR*α* expression	[62]
	High levels of uric acid	Induce the formation of macrophage-derived foam cells and lipid peroxidation	Nrf2/SLC7A11/GPX4 signaling pathway	[63]
	Cigarette smoke extract	Increase PTGS2 expression, GSH depletion, and lipid peroxidation, SMC ferroptosis		[64]

CM death	Models of HF after MI	Downregulate FTH levels, increase oxidative stress and free iron levels, decrease CM viability		[14]
	Erastin, isoprenaline	Increase free iron levels, promote lipid peroxidation, and decrease CM viability		[65]
	Fer-1, puerarin	Inhibit ferroptosis, reduce the loss of CMs	Upregulate the expression of GPX4 and FTH1	[65]
	MI models	Downregulate the levels of GPX4 protein and GPX4 mRNA expression, increase CM death	Reduce GPX4 level	[66]
	HUCB-MSC exosomes	Inhibit H/R-induced CM ferroptosis, attenuate myocardial injury	miR-23a-3p/DMT1 axis	[13]
	Dexmedetomidine	Inhibit ROS production, maintain the structural integrity of mitochondria, inhibit ferroptosis, attenuate myocardial I/R injury	SLC7A11/GPX4 axis	[67]
	Propofol	Reduce SOD and iron accumulation, decrease lipid peroxidation levels, and increase the expression of antioxidant enzymes	AKT/P53 signaling pathway	[68]
	HF models	Downregulate GPX4 and FTH1 protein levels	TLR4-NOX4 pathway	[69]

MF	Inject iron dextran	Increase MDA levels, decrease glutathione peroxidase levels, leading to the occurrence of MF		[70]
	miR-375-3p	Promote MF due to CM ferroptosis	Downregulate GPX4	[71]
	Dexmedetomidine	Inhibit CM ferroptosis after myocardial I/R, reduce the area of MF	SLC7A11/GPX4 signaling pathway	[67]

MH	Apelin-13	Increase iron and ROS levels in mitochondria of CM, induce mitochondrial damage	Induce the expression of SFXN1 and NCOA4	[72]
	Knock out xCT	Increase PTGS2, MDA, and ROS levels, exacerbate Ang II-induced MH	Downregulate xCT	[50]
	Beclin 1 haploinsufficient	Elevate levels of SLC7A11, GPX4, and NCOA4, promote autophagy and ferroptosis, and exacerbate low ambient temperature-induced MH		[73]

## Abbreviations

DNA: Deoxyribonucleic acid
Bcl-2: B cell lymphoma 2
Bax: Bcl-2-associated X protein
mTOR: Mammalian target of rapamycin
ATG: Autophagy-related protein
LC3: Light chain 3
TFEB: Transcription factor EB
DRAM-3: Damage-regulated autophagy modulator 3
NLRP3: NOD-like receptor protein 3
ASC: Apoptosis-associated speck-like protein
IL-1*β*: Interleukin-1beta
IL-18: Interleukin-18
ACSL4: Acyl-CoA synthetase long-chain family member 4
LPCAT3: Lysophosphatidylcholine acyltransferase 3
xCT: Cystine-glutamate antiporter
OxPLs: Oxidized phospholipids
SLC7A11: Subunit solute carrier family 7 member 11
SLC3A2: Subunit solute carrier family 3 member 2
Nrf2: Nuclear factor E2-related factor 2
NCOA4: Nuclear receptor coactivator 4
AA: Arachidonic acid
AdA: Adrenic acid
GCH1: Guanosine triphosphate cyclohydrolase 1
BH4: Tetrahydrobiopterin
CoQ10: Coenzyme Q10
CoQH2: Dihydroubiquione
FSP1: Ferroptosis suppressor protein 1
NADPH: Nicotinamide adenine dinucleotide phosphate
PTGS2: Prostaglandin synthase 2
TLR4: Toll-like receptor 4
AKT: Protein kinase B
HMOX1: Heme oxygenase-1
HUVEC: Human umbilical vein endothelial cells
H/R: Hypoxia/reoxygenation
PTGS2: Prostaglandin-endoperoxide synthase 2.
